This article has been retracted.

# The Tumor Suppressor Role of miR-124 in Osteosarcoma

**DOI:** 10.1371/journal.pone.0091566

**Published:** 2014-06-27

**Authors:** Shuo Geng, Xiaojun Zhang, Jie Chen, Xing Liu, Hepeng Zhang, Xiaoyan Xu, Yan Ma, Baoxin Li, Yunqi Zhang, Zhenggang Bi, Chenglin Yang

**Affiliations:** 1 Department of Orthopedic Surgery, the First Affiliated Hospital of Harbin Medical University, Nangang District, Harbin, Heilongjiang Prov., China; 2 Department of gynaecology and obstetrics, the First Affiliated Hospital of Harbin Medical University, Nangang District, Harbin, Heilongjiang Prov., China; 3 Department of Pharmacology, Harbin Medical University, Harbin, Heilongjiang Prov., China; South China Sun Yat-sen University Cancer Center, China

## Abstract

MicroRNAs have crucial roles in development and progression of human cancers, including osteosarcoma. Recent studies have shown that miR-124 was down-regulated in many cancers; however, the role of miR-124 in osteosarcoma development is unkonwn. In this study, we demonstrate that expression of miR-124 is significantly downregulated in osteosarcoma tissues and cell lines, compared to the adjacent tissues. The expression of miR-124 in the metastases osteosarcoma tissues was lower than that in non- metastases tissues. We identified and confirmed Rac1 as a novel, direct target of miR-124 using prdiction algorithms and luciferase reporter gene assays. Overexpression of miR-124 suppressed Rac1 protein expression and attenuated cell proliferation, migration, and invasion and induced apotosis in MG-63 and U2OS in vitro. Moreover, overexpression of Rac1 in miR-124-transfected osteosarcoma cells effectively rescued the inhibition of cell invasion caused by miR-124. Therefore, our results demonstrate that miR-124 is a tumor suppressor miRNA and suggest that this miRNA could be a potential target for the treatment of osteosarcoma in future.

## Introduction

Osteosarcoma is the most common primary malignant bone tumor with high morbidity in young adults and adolescents [1]. The development of multiple therapeutic strategies for osteosarcoma including wide tumor excision, adjuvant chemotherapy and radiotherapy has significantly improved the prognosis of patients with malignancy [2]. However, 30% of those diagnosed with osteosarcoma do not survive for more than 5 years and approximately 80% of patients eventually develop metastatic disease after surgical treatment, pulmonary metastasis of osteosarcoma patients is the major cause of feral outcome [3], [4].

microRNAs are a class of small non-coding regulatory RNA molecules that exhibit a high degree conservation of structure and function in metazoa [5]. Though miRNAs were first discovered to have crucial functions in Caenorhabditis elegans development, recent progress in cancer biology has shown that miRNAs are frequently dysregulated in diverse cancer subtypes including breast cancer, gastric cancer, lung cancer and hepatocellular carcinoma [6]. To date, miRNAs have been suggested to participate in osteosarcoma development, such as miR-143, miR-31, miR-34 and miR-21 [7]–[10]. However, as only a few miRNAs were reported to be involved in osteosarcoma development, we are still at the beginning of finding the roles of deregulated miRNAs in osteosarcoma carcinogenesis and progression.

Recently, miR-124 has been reproted to be down-regulated in some types of cancer, such as gastric cancer, breast cancer, hepatocellular carcinoma and glioblastoma [11]–[14]. In these malignancies, forced expression of miR-124 inhibits cancer cell growth. However, whether miR-124 is deregulated in osteosarcoma and its roles in osteosarcoma carcinogenesis and progression are still elusive.

In the present study, we found that miR-124 was down-regulated in osteosarcoma cell lines and primary tumor samples, and miR-124 was further identified to be a tumor suppressor, as restoration of miR-124 expression in osteosarcoma cell lines was able to inhibit cell proliferation, promote cell cycle, and suppress cell invasion and metastasis by targeting Rac1. Thus , our date suggest important roles of miR-124 in osteosarcoma pathogenesis and indicate its potential application in cancer therapy.

## Result

### miR-124 is down-regulated in osteosarcoma cell lines and tissues

The expression of miR-124 was examined in 4 human osteosarcoma cells lines (MG-63, U2OS, SOSP-9607, and SAOS-2), 4 osteosarcoma tissues and adjacent non-neoplastic tissues (Fig. 1B). These osteosarcoma cells lines exhibited extraordinarily low expression of miR-124 compared to the 4 pairs of adjacent tissues. Furthermore, the expression of miR-124 in osteosarcoma tissues decreased obviously compared with the adjacent tissues (Fig. 1B).

**Figure 1:** The expression of miR-124 in human osteosarcoma cell lines and tissues. (A) The patient who were diagnosed as in osteosarcoma in H&E staining (original magnification, ×100). (B) The expression of miR-124 in four human osteosarcoma cell lines (MG-63, U2OS, SOSP-9607, and SAOS-2) and four primary tissues (C) and adjacent non-neoplastic tissues (N) using real-time PCR. (C) miR-124 was detected in 70 osteosarcoma patients by real-time PCR. Data is presented as log 2 of fold change of GC tissues relative to non-tumor adjacent tissues. (D) The expression of miR-124 in the osteosarcoma tissues was lower than that in non-tumor adjacent tissues. P<0.01. (E) The expression of miR-124 in the metastases osteosarcoma tissues was lower than that in non- metastases tissues. Experiments were performed three times. All data uses t test and is shown as mean±SD.

### Expression of miR-124 in clinical osteosarcoma patients and their correlation analysis with clinicopathological characteristics

To study the relationship of miR-124 with osteosarcoma development, the expression of miR-124 was detected in 70 clinical patients using Taqman real-time PCR. Out of 70 osteosarcoma samples, miR-124 was down-regulated in 60 cases (60/70, 85.7%) compared with adjacent tissues when the cutoff was set up as 2.0 (Fig. 1C). Meanwhile, miR-124 was up-regulated in 10 cases (10/70, 14.3%). In general, the expression of miR-124 in osteosarcoma tissues was significant lower than in adjacent tissues. (Fig. 1D, p<0.05) The expression of miR-124 in the metastases osteosarcoma tissues was lower than that in non- metastases tissues. (Fig. 1E, p<0.01, independent-samples t test).

### miR-124 inhibits osteosarcoma cell proliferation and cell cycle progression

To study the role of miR-124 in osteosarcoma carcinogenesis, MG-63 and U2OS were transfected with miR-124 mimics, both of them showed great transfection efficiency (Fig. 2A). CCK-8 proliferation assary showed that cell growth rate was reduced in miR-124 mimics-transfected MG-63 and U2OS cells compared with scramble-transfected cells or untreated cells or inhibiors-transfected. (Fig. 2B). To determine if decreased cell viability was a result of cell cycle arrest, we analyzed the cell cycle by flow cytometry. At 48 h post-transfection, miR-124 mimic increased the proportion of MG-63 and U2OS cells in G0/G1-phase and decreased the propotion of MG-63 and U2OS cells in S-phase when compared with the scramble or untreated group. However, miR-124 inhibitor decreased the proportion of MG-63 and U2OS cells in G0/G1-phase and increased the propotion of MG-63 and U2OS cells in S-phase when compared with the scramble or untreated group.

**Figure 2:** Overexpression of miR-124 inhibits osteosarcoma cell growth and affects cell cycle. (A) Expression levels of miR-124 were examined by real-time PCR after transfection of 50 nmol/L of miR-124 mimics or sramble or no transfection or miR-124 inhibitor. (B) Growth of MG-63 and U2OS cells were shown after transfection with 50 nmol/L of miR-10b mimics or sramble or no transfection or miR-124 inhibitor. The growth index as assessed at 0, 24, 48, 72, and 96 hours. (C)The effect of miR-124 on cell cycle progression of MG-63 and U2OS cells after 48-h incubation detected by flow cytometry analysis. Experiments were performed three times. Bars are mean±SD, *p<0.05, **p<0.01 and ***p<0.001.

### miR-124 inhibits cell migration and invasion in vitro

To analyze the role of miR-124 on cell migration and invasion which were the key determinants of malignant progression and metastasis, wound healing and transwell assay were performed in MG-63 and U2OS cells. Both of two cell lines treated with miR-124 mimics were distinctively less migratory than scramble control or untreated cells at 12, 24, and 36 hours after scratching (Fig. 3A). Furthermore, we conducted cell invasion assay of Matrigel and stained the invaded cells to measure the directional invasion ability of the cells after ectopically expressing miR-124 in MG-63 and U2OS cells. The invasiveness of cells transfected with miR-124 mimics was dramatically decreased compared with the scramble control and untreated cells. (Fig. 3B and 3C)

**Figure 3:** Overexpression of miR-124 inhibits osteosarcoma cell migration and invasion. (A) MG-63 and U2OS cells were not transfected or transfected with 50 nmol/L of miR-10b mimics or sramble or inhibitor for 24 hours, and wounds were made. The relative ratio of wound closure per field is shown. (B) (C) MG-63 and U2OS cells were not transfected or transfected with 50 nmol/L of miR-10b mimics or sramble or inhibitor for 24 hours, and migration (B) or transwell invasion (C) assay was performed. The relative ratio of invasive cells per field is shown. Magnification for identification of migration is ×400 and invasion ×40. All data is shown as mean±SD. *p<0.05, **p<0.01 and ***p<0.001.

### miR-124 targets Rac1 in osteosarcoma

As predicted by PicTar, there was complementarity between has-miR-124 and Rac1 3′-UTR (Fig. 4A). MiR-124 overexpression reduced the protein but not the mRNA levels of Rac1 in NP cells. (Fig. 4 B and D). Next, the effect of miR-124 on the translation of Rac1 mRNA into protein was assessed by luciferase reporter assay (Fig. 3C). MiR-124 overexpression remarkably reduced luciferase activity of reporter gene with wild-type, but not mutant Rac 3′UTR, indicating that miR-124 directly targeted Rac 3′UTR.

**Figure 4:** Rac1 is a direct target of miR-124. (A) Predicted duplex formation between human Rac1 3′-UTR and miR-124, Rac1 3′-UTR is highly conserved in different species. Upper panel, sequence alignment of miR-124 with binding site on the Rac1 3′-UTR. Lower panel, sequence of the miR-124 binding site within the Rac1 3′-UTR of four species. (B) MiR-124 cannot alter mRNA level of Rac1 by real-time PCR. (C) Luciferase activity of wild-type (WT-UTR) or mutant (MUT-UTR). (D) Rac1 protein expression in MG-63 cells were transfected with 50 nmol/L of miR-124 mimics , sramble or not transfected.

### Overexpression of Rac1 inpairs miR-124-induced inhibition of invasion in MG-63 cells

To assess the regulation of miR-124 in Rac1 expression, the protein level of Rac1 was analyzed in six miR-124 down-regulated osteosarcoma tissues. Rac1 was up-regulated in five osteosarcoma tissues. (Fig. 5A) We then performed rescue experiments to further validate that.

**Figure 5:** Overexpression of Rac1 inpairs miR-124-induced inhibition of invasion in MG-63 cells. (A) Rac1 is over-expression in osteosarcoma tissues. Western blot analysis of Rac1 protein expression in six patients whose miR-124 expression was down-regulated in osteosarcoma tissues. (B) Overexpression of Rac1 incresed Rac1 protein expression. (C) MG-63 cells were transfected with miR-124 mimics and/or Rac expression vector, and transwell invasion assay was performed. Overexpression of Rac1 inpairs miR-124-induced inhibition of invasion. All data is shown as mean±SD. *p<0.05, **p<0.01 and ***p<0.001.

Rac1 targeting is involved in miR-124–mediated antitumor properties in osteosarcoma cells. Rac1 expression vectors, pcDNA3.0-Rac1 was used to restore Rac1 expression. Inhibition in cell invasion by miR-124–overexpression was significantly attenuated by re-introduction of Rac1 (Fig. 5B).

## Discussion

A large body of evidence has indicated that miRNAs are frequently in a variety of human malignancies [15]. Studies showed a direct link between miRNA function and oncogenesis which is supported by examining the expression of miRNAs in clinical samples [16]. In this study, we found that miR-124 expression is down-regulated in osteosarcoma cells and tissues compared with osteoblastic cell and paired adjacent nontumoral bone tissues. Statistical analyses reveal that the expression level of miR-124 was significantly correlated with the metastases. In addition, we found that overexpression of miR-124 suppressed osteosarcoma cell proliferation, migration and invasion in osteosarcoma cells MG-63 and U2OS. Furthermore, we also identified Rac1 as a direct target of miR-124. Our findings, together with those other groups, suggest that miR-124 has a fundamental role in tumorigenesis and cancer cell invasion.

miR-124 was first demonstrated to be a “brain-specific” miRNA, and was shown to regulate of BDNF [17], [18]. miR-124 also is known to play an important role in the progression of diverse types of cancers [19]–[21]. The expression of miR-124 is very low in many types of cancer cell and miR-124 is usually considered as a tumor-suppressant miRNAs that induces down regulation in many different cancer types, including both solid tumors and hematologic malignancy [22]–[25]. In line with previous studies, in our study, we also found that miR-124 was down-regulated in 60 cases (60/70, 85.7%) osteosarcoma tissues compared with the adjacent tissues and the expression of miR-124 in osteosarcoma tissues was significant lower than in adjacent tissues.

To further verify the role of miR-124 in the development of osteosarcoma, cell transfection was performed. Up-regulation of miR-124 significantly inhibited cell proliferation, migration and invasion; reduced cell viability in osteosarcoma cell lines, indicating that repression of miR-124 might promote tumor progression in osteosarcoma carcinogenesis. Meanwhile, down-regulation of miR-124 significantly promote cell proliferation, migration and invasion; enhanced cell viability in osteosarcoma cell lines, indicating that inhibition of miR-124 might repress tumor progression in osteosarcoma carcinogenesis. These results suggest that miR-124 acts as a tumor-suppressor whose downregulation may contribute to the progression and metastasis of osteosarcoma.

To explore the molecular mechanism by which miR-124 suppressed osteosarcoma cell growth, migration and invasion, we identified Rac1 as a direct target of miR-124 in osteosarcoma cells. This conclusion is supported by the following reasons: complementary sequence of miR-124 is identified in the 3′UTR of Rac1 mRNA; overexpression of miR-124 led to a significant reduction in Rac1 at both mRNA and protein level; miR-124 overexpression suppressed Rac1 3′UTR luciferase report activity and this effect was abolished by mutation of the miR-124 seed binding site. The function of Rac1 is further supported by the observations that inhibition in cell invasion by miR-124–overexpression was significantly attenuated by re-introduction of Rac1. These results indicate that miR-124 may function as a tumor suppressor partly mediated by repressing Rac1 expression in osteosarcoma development.

Rac1 is known to be a member of the Ras superfamily of Rho GTPases, has important roles in cancer invasion [26]–[28]. Rac1 activation is correlated with the progression of many types of cancer such as pancreatic cancer, gastric cancer, and breast cancer [29]–[33]. More investigations have revealed that Rac-dependent cell signaling activation can promote cell adhesion, migration, invasion and metastasis in a variety of cancers, such as prostate cancer, breast cancer, hepatocellular carcinoma, colon carcinoma and renal carcinoma, suggesting that Rac1 plays an important role in tumorigenesis and carcinoma progression [31], [34], [35]. In this study, we confirmed that Rac1 is overexpressed in osteosarcoma. However, the underlying mechanisms are unclear. Our data showed that the ability of miR-124 to target Rac1 may provide one such mechanism of post-transcriptional control of Rac1.

In conclusion, the current study provides novel evidence that miR-124 functions as a tumor suppressor miRNA in osteosarcoma through repression of Rac1 expression. Furthermore, the lower expression of miR-124 in osteosarcoma specimens was correlated with metastasis. Our findings on miR-124 are encouraging and suggest that this miRNA could be a potential target for the treatment of osteosarcoma in future.

## Materials and Methods

### Ethics statement

All patients or patients'parents on behalf of the children agreed to participate in the study and gave written informed consent. This study and consent was approved by the ethical board of the institute of The First Affiliated Hospital of Harbin Medical University and complied with Declaration of Helsinki.

### Patients and tumor samples

Osteosarcoma and their morphologically normal tissues (located >3 cm away from the tumor) were obtained between 2008 and 2012 from 70 osteosarcoma patients undergoing surgery at department of orthopedic surgery, The First Affiliated Hospital of Harbin Medical University. Tissue samples were cut into two parts, one was fixed with 10% formalin for histopathological diagnosis, and the other was immediately snap-frozen in liquid nitrogen, and stored in liquid nitrogen until RNA extraction. None of the patients received radiotherapy or chemotherapy before surgery. The use of the tissue samples for all experiments was approved by all the patients and by Ethics Committee of The First Affiliated Hospital of Harbin Medical University. The characteristics of patients are described in Table 1.

**Table 1:** Clinicopathologic charateristics of patients with osteosarcoma.

Parameter	Total samples	Percentage	miR-124 expression High (n%) Low (n%)		P
Age (years)					0.84
≥13	30	43%	26 (87)	4 (13)	
<13	40	57%	34 (85)	6 (15)	
Gender					0.49
Male	42	60%	35 (83)	7 (17)	
Female	28	40%	25 (89)	3 (11)	
Location					0.31
Femur	40	57%	36 (90)	4 (10)	
Tibia	21	30%	18 (86)	3 (14)	
Humeral bone	6	9%	4 (67)	2 (33)	
other	3	4%	2 (67)	1 (33)	
Pathological facture					0.16
Present	6	8%	4 (67)	2 (33)	
Absent	64	92%	56 (88)	8 (12)	
Metastasis					0.01
Present	10	14%	10 (100)	0 (0)	
Absent	60	86%	50 (83)	60 (17)	
Subtype					0.92
Conventional	29	41%	25 (86)	4 (24)	
Non-conventional	41	59%	35 (85)	6 (15)	

### Cell lines and cell culture

The following human GC cell lines were used in this study: MG-63 (14 years old, male), U2OS (15 years old, female), SOSP-9607(17 years old, male), and SAOS-2 (11 years old, female). These cell lines was purchased from the Cell Resource Center of Institute of Basic Medical Sciences, Chinese Academy of Medical Sciences and Peking Union Medical College (Beijing, China), and was propagated in Dulbecco's modified Eagle medium (Gibco; Invitrogen; Life Technologies, Germany), supplemented with 10% fetal bovine serum (GIBCO, NY, USA) and streptomycin (100 µg/ml), penicillin (100 U/ml).

### Cell transfection

The miR-124 mimics, inhibitor and the scramble mimics, which are non-homologous to the human genome were synthesized by GenePharma (Shanghai, China, Table 2) and transfected into the cells to a final oligonucleotide concentration of 10 nmol/L. All cell transfections were introduced by DharmaFECT1 Reagent (Dharmacon, TX, USA) according to the manufacturer's used instructions. For each cell transfection two or three replication experiments were performed.

**Table 2:** Primer sequence.

Name	Sequence (5′-3′)
miRNA reverse transcription prime	
miRNA-124	CTCAACTGGTGTCGTGGAGTCGGCAATTCAGTTGAGTTGGCATT
U6 snRNA	AAAATATGGAACGCTTCACGAATTTG
Real-time PCR primer sequence	
miRNA-124	TCGGCAGGTAAGGCACGCGGTG
	TCAACTGGTGTCGTGGAGTCGGC
U6 snRNA	CTCGCTTCGGCAGCACATATACT
	ACGCTTCACGAATTTGCGTGTC
GAPDH	AATGGGCAGCCGTTAGGAAA
	TGAAGGGGTCATTGATGGCA
Rac1	GGCTAAGGAGATTGGTGCTGTA
	ACGAGGGGCTGAGACATTTAC

### TaqMan RT-PCR for miRNA expression

Total RNA was extracted from the cells and tissues with Trizol reagent (Invitrogen, Calsbad, CA, USA). MicroRNAs were quantitated by real-time PCR using TaqMan MicroRNA assay (Invitrogen, USA). First-strand complementary DNA (cDNA) synthesis was carried out from 1 µg of total RNA in 12 µl of final volume containing 2 M stem-loop primer, 10 mM dNTP Mix (Invitrogen, USA). The mix was plate at 65°C for 5 min, and then mixed with 5×RT buffer, 0.1 M DTT, 200 U/µl MultiScribe reverse transcriptase and 40 U/µl RNase inhibitor (Invitrogen, USA). The mix was plate at 37°C for 55 min, 70°C for 15 min and then held at −20°C. Real-time PCR was performed using a standard TaqMan PCR protocol. The 20 µl PCRs reactions included 1 µl of RT product, 1 Universal TaqMan Master Mix and 1×TaqMan probe/primer mix (Invitrogen, USA, Table 2). All RT reactions including no-template controls were run in triplicate. All mRNA quantification data were normalized to U6. The relative amount of transcript was calculated using the comparative Ct method.

### Cell proliferation and cycle asssay

Cells were incubated in 10% CCK-8 (Dojindo; Kumamoto, Japan) diluted in normal cultured medium at 37°C until visual color conversion occurred. Proliferation rates were determined at 0, 24, 48, 72, and 96 hours after transfection. Cell cycle analysis was performed on MG-63 and U2OS cell lines 48 hours after transfection. Cells were harvested, washed twice with cold PBS, fixed in ice-cold 70% ethanol, and incubated with propidium iodide (PI) and RNase A, then analyzed by FACS. Each sample was run in triplicate.

### Cell migration and invasion assays

A wound-healing assay was done to assess cell migration. An artificial wound was created 24 hours after transfection using a 200-µL pipette tip on the confluent cell monolayer and mitomyclin C was added to the culture wells. To visualize migrated cells and wound healing, images were taken at 0, 24 and 48 hours.

Invasion assay was evaluated by the ability of cells passing through Matrigel-coated membrane matrix (BD Biosciences). Cells were seeds onto a Matrigel-coated membrane matrix present in the insert of a 24-well culture plate 24 hours after transfection. Fetal bovine serum was added to the noninvading cells were removed. Invasive cells located on the lower surface of the chamber were stained with 0.1% crystal violet (Sigma) and counted.

### Dual luciferase assays

The HEK293T cells were co-transfected with 0.4 µg of the reporter construct, 0.2 µg of pGL-3 control vector, and miR-124 or negative controls. Cells were harvested 24 h post-transfection and assayed with Dual Luciferase Assay (Promega, WI, USA) according to manufacturer's instructions. Firefly luciferase values were normalized to Renilla, and the ratio of Firefly/Renilla values was reported. All transfection assays were carried out in triplicate.

### Western blotting analysis

Western blot analysis was carried out using standard methods. Proteins were separated on 10% SDS-PAGE, and then transferred to PVDF membranes (Amersham, Buckinghamshire, UK). Membranes were blocked overnight with 5% non-fat dried milk and incubated for 2 h with anti-Rac1 antibody (Abcam, England) at 1∶1000 dilution; anti-GAPDH antibody (Proteintech,Chicago, USA) at 1∶50,000 dilution. After washing with TBST (10 mM Tris, pH 8.0, 150 mM NaCl, and 0.1% Tween20), the membranes were incubated for 2 h with goat anti-rabbit antibody (zsgb-bio, Beijing, China) at 1∶5000 dilution and 1∶50000 dilution.

### Rescue assays of Rac1 gene expression

The full length Rac1 cDNAs (which included the ORF and 3′UTR) were PCR amplified and cloned into pcDNA 3.1 to generate the pcDNA-Rac1 constructs, which was used in the rescue assays. MG-63 cells in 6-well plates were first transfected with miR-124 or scrambled dsRNAs (60 nM). After 24 h in culture, these cells were then co-transfected with either miR-124 (20 nM) and 2.0 µg pcDNA-Rac1, miR-124 (20 nM) and 2.0 µg pcDNA-empty. Cells were harvested at indicated time points after hemin addition and assayed as required.

### Statistical analysis

Each experiment was repeated at least three times. Statistical analysis was performed using SPSS 15.0. Data are presented as the mean ± standard deviation. Statistical analyses were done by analysis of variance (ANOVA) or Student's t test and statistical significance level was set at α = 0.05 (two-side).

## References

[1] KobayashiE, HornicekFJ, DuanZ (2012) MicroRNA Involvement in Osteosarcoma. Sarcoma 2012: 359739.2255041910.1155/2012/359739PMC3329862

[2] YangJ, ZhangW (2013) New molecular insights into osteosarcoma targeted therapy. Curr Opin Oncol 25: 398–406.2366647110.1097/CCO.0b013e3283622c1b

[3] OttavianiG, JaffeN (2009) The epidemiology of osteosarcoma. Cancer Treat Res 152: 3–13.2021338310.1007/978-1-4419-0284-9_1

[4] DuongLA, RichardsonLC (2013) Descriptive Epidemiology of Malignant Primary Osteosarcoma Using Population-based Registries, United States, 1999–2008. J Registry Manag 40: 59–64.24002129PMC4476493

[5] GougeletA, PissalouxD, BesseA, PerezJ, DucA, et al (2011) Micro-RNA profiles in osteosarcoma as a predictive tool for ifosfamide response. Int J Cancer 129: 680–690.2094956410.1002/ijc.25715

[6] ChouJ, ShahiP, WerbZ (2013) microRNA-mediated regulation of the tumor microenvironment. Cell Cycle 12.10.4161/cc.26087PMC388563724036551

[7] OsakiM, TakeshitaF, SugimotoY, KosakaN, YamamotoY, et al (2011) MicroRNA-143 regulates human osteosarcoma metastasis by regulating matrix metalloprotease-13 expression. Mol Ther 19: 1123–1130.2142770710.1038/mt.2011.53PMC3129798

[8] van der DeenM, TaipaleenmakiH, ZhangY, TeplyukNM, GuptaA, et al (2013) MicroRNA-34c Inversely Couples the Biological Functions of the Runt-related Transcription Factor RUNX2 and the Tumor Suppressor p53 in Osteosarcoma. J Biol Chem 288: 21307–21319.2372073610.1074/jbc.M112.445890PMC3774399

[9] ZiyanW, ShuhuaY, XiufangW, XiaoyunL (2011) MicroRNA-21 is involved in osteosarcoma cell invasion and migration. Med Oncol 28: 1469–1474.2048026610.1007/s12032-010-9563-7

[10] BaglioSR, DevescoviV, GranchiD, BaldiniN (2013) MicroRNA expression profiling of human bone marrow mesenchymal stem cells during osteogenic differentiation reveals Osterix regulation by miR-31. Gene 527: 321–331.2382745710.1016/j.gene.2013.06.021

[11] XiaJ, WuZ, YuC, HeW, ZhengH, et al (2012) miR-124 inhibits cell proliferation in gastric cancer through down-regulation of SPHK1. J Pathol 227: 470–480.2245065910.1002/path.4030

[12] HanZB, YangZ, ChiY, ZhangL, WangY, et al (2013) MicroRNA-124 suppresses breast cancer cell growth and motility by targeting CD151. Cell Physiol Biochem 31: 823–832.2381685810.1159/000350100

[13] ZhengF, LiaoYJ, CaiMY, LiuYH, LiuTH, et al (2012) The putative tumour suppressor microRNA-124 modulates hepatocellular carcinoma cell aggressiveness by repressing ROCK2 and EZH2. Gut 61: 278–289.2167294010.1136/gut.2011.239145

[14] LvZ, YangL (2013) MiR-124 inhibits the growth of glioblastoma through the downregulation of SOS1. Mol Med Rep 8: 345–349.2381796410.3892/mmr.2013.1561

[15] YatesLA, NorburyCJ, GilbertRJ (2013) The long and short of microRNA. Cell 153: 516–519.2362223810.1016/j.cell.2013.04.003

[16] DassowH, AignerA (2013) MicroRNAs (miRNAs) in colorectal cancer: from aberrant expression towards therapy. Curr Pharm Des 19: 1242–1252.2357005210.2174/138161213804805739

[17] ChandrasekarV, DreyerJL (2009) microRNAs miR-124, let-7d and miR-181a regulate cocaine-induced plasticity. Mol Cell Neurosci 42: 350–362.1970356710.1016/j.mcn.2009.08.009

[18] ZhangJ, LuY, YueX, LiH, LuoX, et al (2013) MiR-124 suppresses growth of human colorectal cancer by inhibiting STAT3. PLoS One 8: e70300.2394055610.1371/journal.pone.0070300PMC3734178

[19] HuntS, JonesAV, HinsleyEE, WhawellSA, LambertDW (2011) MicroRNA-124 suppresses oral squamous cell carcinoma motility by targeting ITGB1. FEBS Lett 585: 187–192.2111232710.1016/j.febslet.2010.11.038

[20] KoukosG, PolytarchouC, KaplanJL, Morley-FletcherA, Gras-MirallesB, et al (2013) MicroRNA-124 Regulates STAT3 Expression and Is Down-Regulated in Colon Tissues of Pediatric Patients With Ulcerative Colitis. Gastroenterology 10.1053/j.gastro.2013.07.001PMC442705823856509

[21] LiKK, PangJC, ChingAK, WongCK, KongX, et al (2009) miR-124 is frequently down-regulated in medulloblastoma and is a negative regulator of SLC16A1. Hum Pathol 40: 1234–1243.1942701910.1016/j.humpath.2009.02.003

[22] LiangYJ, WangQY, ZhouCX, YinQQ, HeM, et al (2013) MiR-124 targets Slug to regulate epithelial-mesenchymal transition and metastasis of breast cancer. Carcinogenesis 34: 713–722.2325091010.1093/carcin/bgs383PMC3581604

[23] LiuK, ZhaoH, YaoH, LeiS, LeiZ, et al (2013) MicroRNA-124 regulates the proliferation of colorectal cancer cells by targeting iASPP. Biomed Res Int 2013: 867537.2369151410.1155/2013/867537PMC3652105

[24] ShiXB, XueL, MaAH, TepperCG, Gandour-EdwardsR, et al (2013) Tumor suppressive miR-124 targets androgen receptor and inhibits proliferation of prostate cancer cells. Oncogene 32: 4130–4138.2306965810.1038/onc.2012.425PMC4111479

[25] FurutaM, KozakiKI, TanakaS, AriiS, ImotoI, et al (2010) miR-124 and miR-203 are epigenetically silenced tumor-suppressive microRNAs in hepatocellular carcinoma. Carcinogenesis 31: 766–776.1984364310.1093/carcin/bgp250

[26] YangQ, LuoGY, LiY, ShanHB, WangHY, et al (2013) Expression of Rac-1 related to tumor depth, lymph node metastasis and patient prognosis in esophageal squamous cell carcinoma. Med Oncol 30: 689.2402665610.1007/s12032-013-0689-2

[27] O'ConnorK, ChenM (2013) Dynamic functions of RhoA in tumor cell migration and invasion. Small GTPases 4.10.4161/sgtp.25131PMC397697024025634

[28] GadeaG, de ToledoM, AnguilleC, RouxP (2007) Loss of p53 promotes RhoA-ROCK-dependent cell migration and invasion in 3D matrices. J Cell Biol 178: 23–30.1760686410.1083/jcb.200701120PMC2064414

[29] BiY, WilliamsJA (2005) A role for Rho and Rac in secretagogue-induced amylase release by pancreatic acini. Am J Physiol Cell Physiol 289: C22–32.1574389010.1152/ajpcell.00395.2004

[30] MatsuokaT, YashiroM, KatoY, ShintoO, KashiwagiS, et al (2011) RhoA/ROCK signaling mediates plasticity of scirrhous gastric carcinoma motility. Clin Exp Metastasis 28: 627–636.2166731110.1007/s10585-011-9396-6

[31] BaugherPJ, KrishnamoorthyL, PriceJE, DharmawardhaneSF (2005) Rac1 and Rac3 isoform activation is involved in the invasive and metastatic phenotype of human breast cancer cells. Breast Cancer Res 7: R965–974.1628004610.1186/bcr1329PMC1410764

[32] ChanAY, ConiglioSJ, ChuangYY, MichaelsonD, KnausUG, et al (2005) Roles of the Rac1 and Rac3 GTPases in human tumor cell invasion. Oncogene 24: 7821–7829.1602772810.1038/sj.onc.1208909

[33] PanY, BiF, LiuN, XueY, YaoX, et al (2004) Expression of seven main Rho family members in gastric carcinoma. Biochem Biophys Res Commun 315: 686–691.1497575510.1016/j.bbrc.2004.01.108

[34] ZavarellaS, NakadaM, BelverudS, ConiglioSJ, ChanA, et al (2009) Role of Rac1-regulated signaling in medulloblastoma invasion. Laboratory investigation. J Neurosurg Pediatr 4: 97–104.1964554010.3171/2009.4.PEDS08322

[35] EngersR, SpringerE, MichielsF, CollardJG, GabbertHE (2001) Rac affects invasion of human renal cell carcinomas by up-regulating tissue inhibitor of metalloproteinases (TIMP)-1 and TIMP-2 expression. J Biol Chem 276: 41889–41897.1155191710.1074/jbc.M105049200

